RETRACTED

# The Role of Computer Remote Monitoring Technology for Nursing Care in Elderly Breast Cancer Complications

**DOI:** 10.1155/2021/5475997

**Published:** 2021-07-15

**Authors:** Ling Wang, Huang Yan, Jing Yan, Liyuan Qian

**Affiliations:** ^1^Department of Nursing, Xiangya Third Hospital, Central South University, Changsha, Hunan 410013, China; ^2^Xiangya College of Nursing, Central South University, Changsha, Hunan 410013, China; ^3^Department of Breast Nail Surgery, Xiangya Third Hospital, Central South University, Changsha, Hunan 410013, China

## Abstract

Geriatric patients undergoing mastectomy have a weakened organism and slow recovery of gastrointestinal function after surgery, which may lead to various complications, affect the absorption of intestinal nutrients, and prolong the healing rate of wounds. Therefore, it is necessary to find an effective nursing program to promote the recovery of gastrointestinal function and prevent postoperative complications in elderly patients undergoing mastectomy. With the continuous development and advancement of computer and communication technologies, telecare is gaining more and more attention and has become an important part of medical information technology construction. Falls endanger the elderly and other special populations, especially after a sudden but unassisted fall, which may be life-threatening. Timely fall detection and rescue can win valuable time for treatment and rescue, which is very important to protect users' health and improve medical monitoring. In order to provide better medical care to the elderly population and reduce the harm caused by falls, this paper will focus on the fall problem of the elderly in telecare. In order to facilitate the detection of falls of the elderly, we design an Android sensor-based data acquisition scheme, using the built-in acceleration sensor in the Android system to collect the human acceleration information, and through the JMS middleware technology, the collected data are transmitted to MATLAB for analysis and processing in real time. This paper preprocesses and synthesizes the collected human body data and visualizes the acceleration changes of various typical daily activities of the human body and breast cancer, then extracts the relevant data features according to the synthesized SVM curve, constructs a pattern recognition algorithm using the extracted features, and verifies the effectiveness of the pattern recognition algorithm through experiments.

## 1. Introduction

In recent years, with the continuous development and progress of society, the accumulation of social wealth, the significant improvement of people's material living standards, and the progress of national awareness, more and more people are concerned about their health status [1]. However, the increasing work pressure, deteriorating living environment, and decreasing exercise have led to the decrease of the overall health level of citizens nowadays. With the development of computer and communication technology, telecare has been developed rapidly, and people can test their health condition at home and communicate with medical personnel through computer, which not only can detect some potential diseases in time but also reduce the burden of patients' families [2]. With the continuous development and progress of society and people's consciousness, population aging has become a major problem faced by all countries in the world [3].

RETRACTED

According to the sixth national census, as of 2010, the population aged 60 years and above reached 178 million, accounting for 13.26% of the total population, compared with 10.33% in 2000, an increase of 2.93 percentage points from the previous year [4]. Among them, the elderly population aged 65 and above reached 119 million, accounting for 87% of the total population, up 1.19 percentage points from the 2000 census, far higher than the standard line of 7% defined by the United Nations for an aging society [5]. According to the latest statistical results published by the National Bureau of Statistics, the aging population in China has reached 200.2 million people at this stage. According to various statistics, China has entered the aging society since 2000, and the aging process of China's society has been deepening in the last decade [6–8]. The implementation of family planning policies in China has led to a significant decrease in the number of newborns, coupled with the fact that the values of the Chinese people have changed significantly, and the structure of families tends to be smaller, with children preferring to live separately from their parents [9]. As a new medical model, it is widely used in various medical fields such as telemedicine education, telemedicine, and telehealth. Telemedicine systems not only save patients money on medical costs but also have a very positive effect on the detection and treatment of diseases such as many chronic diseases. Nowadays, population mobility is more frequent than before, and more young people are moving to big cities, leaving little time for their families, resulting in an increasing number of “empty nest families” [10]. The aging of the population has become a serious social problem, and the problem of “empty nest families” has increased people's concern about the elderly, which has led to the problem of health care for the elderly [11–13]. In the above-mentioned social context, the health of the elderly has become one of the most important issues to be solved in today's society [14]. Nowadays, the demand for medical equipment for the elderly is increasing year by year. In the traditional guardianship mode, the elderly need to be sent to the hospital, and then with the help of the testing equipment in the hospital, the physical examination is carried out, and then the diagnosis report is issued by the doctor, and sending the sample not only brings great inconvenience to the patient's life but also brings expensive economic pressure [15–17]. With the continuous development of computer and communication technology, a new medical care model of telecare delivery has emerged, which can well solve the shortcomings of the traditional model and bring real-time telecare services to users.

RETRACTED

Therefore, the study of elderly breast cancer complications detection in telecare highlights its important practical significance. If a breast cancer detection system that is easy to carry, accurate in detection, and timely in judgment can be developed, which can provide timely detection of breast cancer and can send out help information at the first time, on the one hand, it can win precious time for treatment and rescue and reduce many unnecessary losses, which is on the other hand, it can improve the quality of life of the elderly, enhance their ability to live independently, provide real-time protection for their health, and reduce the burden of their families and society. Program nursing is a kind of care that combines modern communication, computer and modern medicine and other advanced technology means, disease diagnosis, and treatment for the purpose of providing remote medical assistance services for patients. The continuous development of modern computer and communication technology and the application of more and more new technologies have gradually brought telecare into the sight of the general public, and its service model has been developing and improving. In particular, with the spurt of mobile Internet and new concepts such as Internet of Things and cloud computing, more and more research institutions and scholars are paying attention to telecare and continuously enriching the discipline of telecare to make it more efficient, humane, and intelligent. From these, the forward fall appears at two different peaks, the first peak is slightly lower than the second, and by intuitive judgment of the fall position we can see that the first peak is caused by the human knee touching the ground, and the second occurs when the entire body touches the ground, two peaks appeared during weightlessness.

## 2. Telecare of Complications

### 2.1. Related Theories and Key Technologies

The main purpose of telecare is to provide users with timely and effective remote monitoring services using telecommunication technology and computer technology, to provide users with medical assistance guidance, and to send alerts to relevant medical institutions or relatives of the monitored person when an unexpected condition is detected. In this chapter, we will introduce the theory of remote care and breast cancer detection and introduce the Android platform technology used in the system development. Telecare incorporates sensor technology, fluency technology, information technology, and nursing care and other related technologies to provide telemedicine information and services through the transmission of data, video, audio, or image information and is not limited by geographic location or time and space. In a broad sense, telecare uses telematics and computer technology to achieve remote transmission, analysis, and storage of electronic medical data, thus realizing various medical functions such as daily health monitoring, disease treatment, and health care.

RETRACTED

As a new medical model, it is now widely used in several medical fields, such as telehealth education, telesurgery, and teleconsultation. Telecare systems not only save patients' care costs but also have a very positive effect on the detection and treatment of many chronic diseases. Through this system, remote care and monitoring for the elderly can be realized, and the elderly can always maintain effective information communication with distant medical institutions and doctors, which provides great medical health protection for special groups such as the elderly. The system implementation of remote care is mainly divided into H parts, as shown in Figure 1, which are user terminal, communication network, and remote care supervision platform.

The user terminal is mainly responsible for collecting blood pressure, body temperature, pulse rate, blood glucose concentration, blood oxygen concentration, motion acceleration, and other human characteristics data and then sending the collected data to the remote care supervision center through network communication, and the supervision center also gives medical advice to the patient through the analysis and processing of data and sends timely medical advice to the medical institution or the patient's family when special conditions are found in the monitored person. In the user layer, since the acceleration of the normal body in daily life and the acceleration of the body under abnormal conditions such as falls are very different, it is available to determine whether there is a fall by analyzing related information such as acceleration.

RETRACTED

Telecare has a good effect on the daily care of chronic diseases such as cerebrovascular diseases and unexpected events such as dirty diseases and breast cancer in the elderly. Its biggest advantage is that it can achieve efficient resource sharing, provide timely emergency assistance, provide real-time security for the monitored person, and effectively save hospital and patient expenses.

### 2.2. Detection Fundamentals

Breast cancer patients often suffer from complications such as dizziness and fainting, which subsequently bring about fall injuries and other challenges. The next example of fall detection is illustrated. A fall usually refers to a sudden, uncontrolled change in body position, usually resulting in an uncontrolled fall onto a relatively low object such as the ground or stairs, but the cause of a fall does not include spleen, healing pain, or a knock from external violence. Falls can cause great damage to the human body and may result in fractures, induce vascular diseases, tissue contusions, and other accidental injuries, so falls should be taken seriously enough. There are many causes of falls, which are summarized in this branch classification.

#### 2.2.1. Age Factor

Falls mostly occur in the elderly and have the highest probability of causing accidental injuries. The reason is that the skeletal and muscular system of the elderly degenerates and the absorption capacity of the trace elements required by the human body becomes weaker, resulting in symptoms such as osteoporosis and weakening of the lower limbs. In addition, the elderly are more reactive and less flexible than young people, and their ability to control the body's dynamic balance is also greatly reduced. The decline in all physical indicators leads to changes in gait of the elderly, the pace of walking becomes smaller, and the swing of the arms is reduced, thus causing instability of the body weight. According to the statistics of 110 patients admitted to a hospital from 2011 to 2013, there were 60 male patients and 50 female patients, and 80 patients over 60 years old, accounting for 73% of all patients. From this, it can be found that the probability of falling increases sharply in elderly people because of their age.

#### 2.2.2. Environmental Factors

The environment is an important factor that causes frequent falls in the elderly. When a person is in a poor environment, the probability of having a fall increases significantly. For example, if the lighting in the stairway corridor is poor, it is easy to fall when going up and down the stairs because you cannot see the steps. The endurance means the skeletal and muscular system of the elderly degenerates, and the absorption capacity of the trace elements required by the human body becomes weaker. A large number of statistical studies have shown that the probability of falling is much greater outdoors than indoors. The outdoor environment is relatively complex and people may not be able to adapt quickly to the environment, so they are prone to falls and other unexpected situations.

RETRACTED

#### 2.2.3. Social Factors

Older people generally have higher self-esteem, are afraid of causing trouble to others, and like to live independently, as shown by the fact that older people generally do not obey old age, think they can do a lot, and overestimate their own physical state and fitness state, which often leads to the occurrence of accidental falls. In addition, such as anxiety and other factors may also reduce the sensitivity of the elderly to the environment, many risk factors are not eliminated in time, resulting in the occurrence of falls.

#### 2.2.4. Disease and Drug Factors

The elderly are generally weaker and more susceptible to disease, so most of them will need to take long-term drugs to control the development of their condition. However, many medications can affect the body's vision, blood pressure, and mind, which in turn affect people's control of their bodies, thus increasing the probability of falls occurring. For example, certain sedative and sleep-aid medications can affect the body's control of its own balance.  Figure 2 shows a statistical table of the causes of complications in a hospital survey of 100 elderly patients, from which it can be seen that there are various factors that trigger complications in the elderly, but the most important causes are focused on the weakening of the elderly, diseases, and the environment in which they are located as a danger.

There are various causes of human falls, but falls are generally accompanied by changes in human posture and position. The main postures of the human body in daily life can be classified from static and dynamic:

1. The user terminals collect mainly human data such as blood pressure, body temperature, pulse rate, blood sugar levels, blood oxygen concentration, and motor acceleration
2. Then, they transmit the collected data via network-controlled information to the Telemedicine Monitoring Centre, and the monitoring body advises patients by analyzing and processing the data medically
3. And if a particular disease is found in the monitored compartment, send timely medical advice to medical institutions or patients' families

Among them, the elderly are mostly static and slow dynamic movements in their lives, and the movements of going up and downstairs, lying down, and sitting down are also relatively slow, and they rarely engage in strenuous running and other activities. Therefore, the detection of abnormal behaviors such as falls in the elderly should be based on the characteristics of the elderly population, which are different from those of children and young people. The relatively strenuous activities in the daily life of the elderly generally include going up and downstairs and jogging. Therefore, in the study of falls in the elderly, these activities should be focused on the study of falls usually occurring within a very short period of time; according to the data on fall behavior research, the human body generally falls between 1 s and 3 s during the whole process of falling. When the body is standing normally, the force by the ground is stable; when the body is out of balance and in a weightless state, the force by the ground will be rapidly reduced; when the body is in contact with the ground collision, the force will be a sharp change; when the body is at rest at the end of the fall, the force is in a stable state. This can be roughly divided into four stages of the process of human falls.

RETRACTED

In the first stage, the human body is in a normal standing state. At this time, the human body is affected by gravity and ground force to maintain stability; the human body at this time by the force of the ground remains in a stable state, and at this time the body's acceleration in all directions also remains basically stable.

In the second stage, the body falls, the body tilts, but the body does not have a large area of direct contact with the ground. At this time, the human body will appear tilted weightlessness, as shown by the rapid reduction of the force of the ground on the human body, the acceleration in all directions obviously changes.

Third stage: the human body after a fall and the ground and other contact collision stage. As the human body falls, and falls generally occur in a very short period of time, the human body is difficult to make self-protection, as a result the human body will have a violent collision process with the ground, and there will be a repeated process; the ground force at this stage is an undulating process, rapidly increases, and then will quickly reduce, and several fluctuations in the process of amplitude will gradually reduce.

Fourth stage: the resting stage after a fall. When a fall occurs, the human body will generally have a relative stationary phase, and if the fall is serious, it may lie on the ground for a while. This process is due to the body lying flat on the ground, so the force on the ground by the body in this process is also smooth.

The acceleration of the human body in normal activities in daily life and the acceleration of the human body in abnormal conditions such as falls are significantly different, so the acceleration and other related information can be analyzed to determine whether the human body has fallen—data analysis.

RETRACTED

### 2.3. Remote Monitoring Based on Android Platform

The Android system has a wealth of built-in sensors, so data can be collected, analyzed, and communicated with Android mobile terminals. Android was chosen because of the following reasons.

First, the Android system is open source, and it is easy to understand the overall architecture of the Android system in detail, and the values of the parameters inside the Android system can be modified as needed.

Second, Android has strong application layer developability; the system provides a rich API; according to the need, optimize the system operation interface to achieve data collection, data analysis, abnormal SMS alarm, user information settings, and other functions.

Third, the Android system supports GPRS, IFI, Bluetooth, AP hotspot, and other network types, and its powerful network function can ensure the reliability and stability of data transmission of the remote care system; and fourth, with the continuous popularity of smart phones, the Android system with its good user experience and relatively low price gradually becomes the trickster among all intelligent systems, occupying the majority of user groups.

In summary, this paper selects the Android system mobile device as the personal terminal of fall detection system. The Android system architecture adopts a layered structure design, which is divided into four layers, from high to low: application layer, application framework layer, system runtime library layer, and Linux kernel also called layer P. Its detailed system framework is shown in Figure 3.

There are many kinds of human parameters that need to be measured in telecare, such as body temperature, blood saturation, electricity, pulse, respiration, and movement status. Different signals require different acquisition devices and acquisition methods. Through the analysis and introduction in the previous chapters, we know that the information of human body acceleration can reflect whether the human body is in the normal activity state or in the special condition such as fall, so we need to acquire the relevant human body data. Convenient and intelligent perception of the surrounding environment, its lightweight, and intelligent features are also very suitable for remote control, so this chapter will focus on using the built-in acceleration sensor in the Android system to obtain the acceleration information of the human body. Nowadays, smart phones have long become an indispensable part of people's daily life, and a lot of information exchange is also done based on hand, and cell phones have gradually developed from blue-screen and color-screen phones that could only make phone calls and send text messages to smart phones with high screen resolution, superior performance, and more and more complete functions. In fact, the general smart phones now have many built-in sensors, i.e., most smart phones are equipped with acceleration sensors, gravity sensors, pressure sensors, rotation vector sensors, gyroscope sensors, etc. These built-in sensors can provide data well and accurately, so the smartphone can be selected as the data acquisition device for the fall detection system in this paper. The main parameters of the cell phone selected in this paper are as follows: the system version is Android0S4.3; the CPU is Qualcomm Snapdragon 800 (MSM827); and the built-in acceleration sensor model is LIS3DH3-axis, which is produced by STMicroelectronics and has the advantages of low power consumption and small size. Advantages: very suitable for motion-sensitive occasions or motion space is relatively limited, and the power consumption requirements of low occasions, in ±2g, ±4g, ±8g, ±16g of the full range, have good stability and accuracy, and the accelerometer chip has a built-in temperature sensor and H-way analog-to-digital converter and can be simply integrated with accompanying chips such as gyroscopes to achieve various functions such as motion data measurement and 4D/6D direction detection. The main functional characteristics of the acquisition device and the H-axis acceleration sensor LIS3DH are shown in Figure 4.

RETRACTED

The data acquisition is mainly done by acquiring the accelerometer data from the phone through the acquisition program. The system interface wraps the acceleration sensor and provides a sensor class that can get the required value according to the type of sensor. Since the sensor values are frequency-based and return a value every fixed time, a trigger mechanism is needed to listen to the sensor with events. Whenever the accelerometer detects a change in the accelerometer, a sensor event is generated. A sensor event is an object from which the program gets the acceleration value.

## 3. Results and Analysis

### 3.1. Implementation of Pattern Recognition

For the collected data simulating the fall and daily activities of the elderly, the corresponding data processing and analysis are performed with the help of the machine, and then certain features in the data are extracted and used to make judgments on human activity patterns such as falls, so as to establish a human fall detection model. The main steps are divided into four parts: acquisition of information, preprocessing of data, extraction and selection of data features, and classification of classifier, and its pattern recognition process is shown in Figure 5.

1. The observation object, i.e., the input object of the needed information. In this paper, we focus on the fall detection of the elderly in telecare, so the observation objects are mainly for the elderly.
2. Data acquisition is mainly self-developed data acquisition program, based on Android sensors for data acquisition, and then through the set data acquisition scheme, the Android sensors collected human acceleration and other information transmitted to the computer, the computer will store the data, and the implementation of this part has been explained in the previous chapter.
3. Data preprocessing is mainly to filter out the interference and noise in the process of information acquisition and to smooth the obtained data to a certain extent as much as possible without changing the characteristics of the data.
4. Selection and extraction of data features. Since the amount of acquired information data is generally large, in order to be able to quickly complete the entire process of classification and identification, it is necessary to analyze and process the data, and then extract the features that best reflect the characteristics of the data, and then compose a data feature vector set from these data features and conduct research on these feature vector sets.
5. Classifier selection. A set of pattern discrimination algorithms is designed for the features of the acquired data, and the patterns with recognition are assigned to their respective corresponding pattern classes. The classifier is trained with a certain number of training samples to derive a set of classification discriminant rules, which can classify the behavior to determine whether a fall has occurred.
6. Classification decision. It mainly uses the above extracted classification discriminative rules to classify the recognized patterns accordingly and then output the classification discriminative results.
7. Testing stage. The test samples are subjected to corresponding data preprocessing, feature extraction, and classification decision processes, and then the classification results are output, and then the test samples are compared to check the effectiveness of the classification discriminant rules, and the corresponding corrections are made for the deficiencies in them.

RETRACTED

Usually, the acceleration signal obtained from the human body is superimposed by the human motion acceleration component, the human body gravitational acceleration component, the human body's own jitter, and the system measurement noise of a variety of signal quantities, and there will be a large number of spike pulses and other noise in the signal. If the analysis is performed directly on the acquired data, the noise may affect the analysis results, so it is necessary to filter and denoise the original signal output from the acceleration lift. In this paper, the median filter is selected for noise reduction. The median filter median is the sample value in the sampling sequence where the value is greater than half of the sample value and less than the other half. Therefore, when processing the signal, the sampling sequence is first sorted and then the middle value is taken out. The median filter is a nonlinear filtering signal processing technique whose main principle is to use a window of a given length to cross the original signal sequence in turn, replacing the sample value centered in the window with the median value of the signal sequence contained in that window. Suppose there is a sequence of

(1) $$\begin{array}{c} F:∼\sum_{i=0}^{n}\left\{f_{1},f_{2},f_{3},\ldots ,f_{n}\right\}, \end{array}$$

a window of odd *m* length is selected, and then this sequence is median-filtered. First, *m* consecutive numbers are drawn from the sequence:

(2) $$\begin{array}{c} F:∼\sum_{i=0}^{n}\left\{f_{1-k},f_{2-k},f_{3-k},\ldots ,f_{n-k}\right\}. \end{array}$$

Among them,

(3) $$\begin{array}{c} k=\frac{m+1}{2}. \end{array}$$

Then, the *m* points are sent to be sorted by the magnitude of the values, and their middle values are taken as the filtered output, and the expressions are

(4) $$\begin{array}{c} F=\frac{\sum_{i=0}^{n}\left\{f_{1-k},f_{2-k},f_{3-k},\ldots ,f_{n-k}\right\}}{\text{med}\left(m+1\right)}. \end{array}$$

In this paper, the size of the median filter window is chosen to be 3. Experiments have shown that when *n* is chosen too large, the effect becomes relatively poor. After using the median filter to filter the collected data, the signal of acceleration is worth to a certain smoothness, and the purpose of filtering noise is achieved. The acceleration curves of human motion after data preprocessing are shown in Figure 6.

The direction of the H-dimensional vectors *X*, *Y*, and *Z* of the acceleration sensor is closely related to the direction of the device, and different directions can cause significant differences in the H-dimensional vector data. Therefore, it is common to use the synthetic processing of 3D acceleration to eliminate the influence of direction. The H-dimensional acceleration is synthesized by using the previously constructed human coordinate system and the acceleration synthesis formula, i.e., at a certain time *t*, the synthesized acceleration is

(5) $$\begin{array}{c} \tilde{a}=\sqrt{\left(x^{2}+y^{2}+z^{2}\right)},\\ Fa=\sqrt{\frac{\sum_{i=0}^{n}\left\{f_{x},f_{y},f_{z}\right\}}{\text{med}\left(m+1\right)}}. \end{array}$$

This method is called SVM (signal vector magnitude) eigenvolume method. Because in the process of human motion, it is impossible to predict the change of weight and direction, and SVM is the magnitude of the synthetic acceleration vector of the three axes of acceleration, which is not related to the direction of human motion but only reflects the sharpness of the change of human velocity, and SVM is larger when the change of human motion velocity is sharp, and vice versa is smaller, so the influence brought by the direction of human motion can be avoided with SVM. A section of the data of going downstairs, for example, after data synthesis, the SVM curve of going downstairs is obtained as shown in Figure 7.

RETRACTED

It can be seen from the figure that the general direction of the SVM curve after the synthesis formula is basically the same as before the synthesis, which eliminates the influence of the direction and can well represent the change of the human body's movement speed. Nowadays, most fall detection systems use a variety of different threshold values of eigenvalues to synthesize the determination and improve the accuracy of fall detection. In the previous section, this paper placed the acquisition device on the waist of the experimenter, so for the selection of the fall feature vector, the specificity of the change of human waist posture should also be considered. The feature extraction method uses the commonly used confusion window method, which can make the length of acceleration signal shorter and adjust the length of different action acceleration signals.

SVM top is the peak of the SVM curve, which is also the peak of the synthetic acceleration curve, and can be used to reflect the dramatic degree of signal change at a certain moment. During a fall, the larger the SVM top is, the more dramatic the change in acceleration is, and the more dramatic the change in human posture can be assumed to be. Therefore, a threshold value can be set, and when the SVM top exceeds this threshold value, it is determined that a suspected fall may occur at this time, and the data near this peak are focused on the analysis. As shown in Figure 8, the SVM changes dramatically when the human body falls in either direction. The most obvious change is to the right, with a maximum value of more than 5g; although the front, back, and left changes are not so obvious, they also reach or exceed 4g. Because there is a sense of self-protection during the data collection process, pad protection may weaken the monitoring effect. Among them, the forward fall appeared at two different peaks, the first is a little lower than the second; and through the intuitive judgment of the fall position, we can know that the first peak is generated by the human knee contact with the ground and the second is generated by the entire body contact with the ground; the two peaks appeared between the weightlessness.

RETRACTED

As can be seen from the SVM plot of fast walking in Figure 9, both walking and fast synthetic acceleration have obvious periodic characteristics, and both SVM curves show a certain oscillation, but the amplitude of the oscillation is significantly smaller than that of stepping down, where the maximum value of SVM for walking is generally around 2g, and fast walking is also under 3g, and both are accompanied by a phase of weightlessness.

In summary, get the human body daily activities in the synthetic acceleration maximum as shown in the table above; when the human body is usually stationary, standing, SVM will be in a relatively stable state, about Ig, and there will not appear a wide range of fluctuations in SVM; when the human body is in a fast walking state, certain fluctuations will appear in SVM, but the overall fluctuations are not very large, generally within 3g; when in the sitting or standing state, SVM fluctuations are not obvious, only slight fluctuations, generally within 2g; and when running and other strenuous exercise, violent fluctuations will appear in SVM, generally to be in the range of 4g–6g, and this good change is relatively already very obvious.

During the nonstrenuous movements such as fast walking, sitting down, standing up, running, and other normal activities in daily life, excluding running, the combined acceleration does not exceed 3g, but the synthetic acceleration varies greatly when running and may be between 4g and 6g depending on the degree of strenuousness; the elderly mainly perform nonstrenuous movements in daily life, so those strenuous and special movements will not be the focus of the study. Through the above study, the overweight threshold was set to 33 because the movements of the elderly in normal life such as sitting, walking, going up, going down, and squatting are slow, and the synthetic acceleration is generally under 3 g, only the special strenuous activities such as running may exceed the set overweight threshold, so the characteristic value can effectively distinguish most of the falls from nonfalls.

## 4. Conclusion

In this paper, we conducted a study on breast cancer complications in elderly people in telecare and constructed a telecare system based on Android fall detection to alleviate the current situation of poor health protection for the elderly population due to the aging of society. The system can detect the activities of the elderly by analyzing and extracting their daily activity characteristics data and provide remote alarm service when danger is detected and then take corresponding rescue measures. This paper addresses the shortage of no real fall data for research, designs its own data collection program based on Android devices, and proposes a real-time data transfer method between Android and MATLAB using JMS middleware, transfers the data collected by Android in real time, makes full use of MATLAB ready-made algorithm toolkit, and constructs an intelligent system. The data analysis and modeling environment based on mobile devices and the MATLAB server is constructed as a simulation environment for pervasive computing. This paper designs the overall architecture of the Android-based fall detection telecare system and analyzes and designs each functional module of the personal monitoring terminal to realize the whole system process from data collection to alarm information release. And for the characteristics of the mobile terminal system, the low-power museum research is conducted to improve the practicality of the system. In the future, you can set a threshold value, and if the SVM peak exceeds that threshold, you will find that there may be a suspicious decrease at that time and the data close to that peak will be analyzed.

RETRACTED

## Figures and Tables

**Figure 1:** Telecare system implementation diagram.

**Figure 2:** Breast cancer complication statistics.

**Figure 3:** Android-based system detection architecture.

**Figure 4:** Device detection functions and features.

**Figure 5:** Pattern recognition flowchart.

**Figure 6:** Acceleration data curve after filtered fall.

**Figure 7:** Synthetic acceleration SVM curve.

**Figure 8:** Falling SVM curve.

**Figure 9:** SVM curves for normal walking and fast walking.

## Data Availability

Data sharing is not applicable to this article as no datasets were generated or analyzed during the current study.

## References

[1] Rubin G. D., Ryerson C. J., Haramati L. B. (2020). The role of chest imaging in patient management during the COVID-19 pandemic: a multinational consensus statement from the Fleischner society. *Chest*.

[2] McGonagle D., Sharif K., O’Regan A., Bridgewood C. (2020). The role of cytokines including interleukin-6 in COVID-19 induced pneumonia and macrophage activation syndrome-like disease. *Autoimmunity Reviews*.

[3] Zhou X., Snoswell C. L., Harding L. E. (2020). The role of telehealth in reducing the mental health burden from COVID-19. *Telemedicine and E-Health*.

RETRACTED

[4] Lurie N., Carr B. G. (2018). The role of telehealth in the medical response to disasters. *JAMA Internal Medicine*.

[5] Cheng V. C.-C., Wong S.-C., Chuang V. W.-M. (2020). The role of community-wide wearing of face mask for control of coronavirus disease 2019 (COVID-19) epidemic due to SARS-CoV-2. *Journal of Infection*.

[6] Staffell I., Scamman D., Velazquez Abad A. (2019). The role of hydrogen and fuel cells in the global energy system. *Energy & Environmental Science*.

[7] Gielen D., Boshell F., Saygin D., Bazilian M. D., Wagner N., Gorini R. (2019). The role of renewable energy in the global energy transformation. *Energy Strategy Reviews*.

[8] Ahmed E., Yaqoob I., Hashem I. A. T. (2017). The role of big data analytics in internet of things. *Computer Networks*.

[9] Hope M. D., Raptis C. A., Shah A., Hammer M. M., Henry T. S. (2020). A role for CT in COVID-19? What data really tell us so far. *The Lancet*.

[10] Li Y., Xia L. (2020). Coronavirus disease 2019 (COVID-19): role of chest CT in diagnosis and management. *American Journal of Roentgenology*.

[11] Bancerek G., Byliński C., Grabowski A. (2018). The role of the Mizar mathematical library for interactive proof development in Mizar. *Journal of Automated Reasoning*.

[12] Roberge S., Nicolaides K., Demers S., Hyett J., Chaillet N., Bujold E. (2017). The role of aspirin dose on the prevention of preeclampsia and fetal growth restriction: systematic review and meta-analysis. *American Journal of Obstetrics and Gynecology*.

[13] Sproston N. R., Ashworth J. J. (2018). Role of C-reactive protein at sites of inflammation and infection. *Frontiers in Immunology*.

[14] Malakayev S., Aralbaev R. (2019). Early complications after surgical treatment of breast cancer in the elderly and senile. *Bulletin of Science and Practice*.

[15] Vologdina I. V., Poroshina E. G., Zhabina R. M., Stanzhevsky A. A. (2019). Prevalence of risk factors of cardiovascular complications in elderly women with left breast cancer. *HERALD of North-Western State Medical University named after I. I. Mechnikov*.

[16] Losada B., Guerra J. A., Malón D., Jara C., Rodriguez L., Del Barco S. (2019). Pretreatment neutrophil/lymphocyte, platelet/lymphocyte, lymphocyte/monocyte, and neutrophil/monocyte ratios and outcome in elderly breast cancer patients. *Clinical and Translational Oncology*.

[17] Hershman D. L., Till C., Wright J. D. (2019). Association of baseline cardiovascular risk factors and health care utilization and costs in elderly breast cancer patients enrolled in SWOG clinical trials. *Journal of Clinical Oncology*.

